# Multi-Level Interactions between the Nuclear Receptor TRα1 and the WNT Effectors β-Catenin/Tcf4 in the Intestinal Epithelium

This article has been retracted.

**DOI:** 10.1371/journal.pone.0034162

**Published:** 2012-04-03

**Authors:** Maria Sirakov, Seham Skah, Imtiaz Nisar Lone, Julien Nadjar, Dimitar Angelov, Michelina Plateroti

**Affiliations:** 1 Institut de Génomique Fonctionnelle de Lyon, Lyon, France; 2 Laboratoire de Biologie Moléculaire de la Cellule, Université de Lyon, Université Lyon 1, Ecole Normale Supérieure de Lyon, Lyon, France; National Cancer Center, Japan

## Abstract

Intestinal homeostasis results from complex cross-regulation of signaling pathways; their alteration induces intestinal tumorigenesis. Previously, we found that the thyroid hormone nuclear receptor TRα1 activates and synergizes with the WNT pathway, inducing crypt cell proliferation and promoting tumorigenesis. Here, we investigated the mechanisms and implications of the cross-regulation between these two pathways in gut tumorigenesis *in vivo* and *in vitro*. We analyzed TRα1 and WNT target gene expression in healthy mucosae and tumors from mice overexpressing TRα1 in the intestinal epithelium in a WNT-activated genetic background (*vil*-TRα1/Apc mice). Interestingly, increased levels of β-catenin/Tcf4 complex in tumors from *vil*-TRα1/Apc mice blocked TRα1 transcriptional activity. This observation was confirmed in Caco2 cells, in which TRα1 functionality on a luciferase reporter-assay was reduced by the overexpression of β-catenin/Tcf4. Moreover, TRα1 physically interacted with β-catenin/Tcf4 in the nuclei of these cells. Using molecular approaches, we demonstrated that the binding of TRα1 to its DNA target sequences within the tumors was impaired, while it was newly recruited to WNT target genes. In conclusion, our observations strongly suggest that increased β-catenin/Tcf4 levels i) correlated with reduced TRα1 transcriptional activity on its target genes and, ii) were likely responsible for the shift of TRα1 binding on WNT targets. Together, these data suggest a novel mechanism for the tumor-promoting activity of the TRα1 nuclear receptor.

## Introduction

The intestinal epithelium is a dynamic tissue that is continuously renewed through stem cells and committed progenitors, located in the crypts of Liberkün [1], [2]. The balance between proliferation and differentiation in the crypts is maintained by the fine cross-regulation among several pathways, including WNT, Hedgehog, Notch, BMP, and thyroid hormones (THs) [3]–[6]. These pathways are key players of intestinal homeostasis, and their deregulation is correlated with the onset of colorectal cancer [7]–[9]. The molecular basis of their action is only partially understood, and the mechanism of cross-regulation that occurs between these signaling pathways is still a puzzle. We previously demonstrated that TH signaling in the mouse intestine is involved in development, homeostasis and cancer susceptibility [10]#. THs act through nuclear hormone receptors, the TRs, which are encoded by *THRa* and *THRb* loci [11]. These transcription factors activate or repress the transcription of target genes by binding to specific DNA sequences called thyroid hormone response elements (TREs) [12], and they are involved in several cellular responses, such as cell proliferation, cell differentiation and apoptosis [5], [13]. TH signaling in the mouse intestine is mediated by TRα1, given that TRα^0/0^ [14] mice as well as hypothyroid mice have reduced cell proliferation in the crypts during development and in adulthood [15]. Recently, we showed that the constitutive TRα1 overexpression in the intestinal epithelium (*vil-*TRα1 mice) allows increased cell proliferation and adenoma development; this overexpression also enhances the intestinal tumorigenic process in an Apc mutated genetic background (*vil-*TRα1/Apc^+/1638N^ mice) [9]. Interestingly, one of the molecular features of the *vil*-TRα1/Apc mice is the increased activity of the WNT pathway compared with that of the Apc mutants [9]. This is in agreement with our previous studies showing that TRα1 activates the WNT pathway *via* the transcriptional regulation of the genes *Ctnnb1* and *Sfrp2* [15], [16].

β-Catenin, the protein encoded by *Ctnnb1*, was originally identified as a structural component of cell adhesion complexes [17]. Upon increased cellular levels and nuclear accumulation, β-catenin interacts with transcription factors of the T-cell factor (Tcf) and lymphocyte-enhancer factor (Lef) families [18]. β-catenin/Tcf-Lef complexes are the downstream molecular effectors of the WNT signaling pathway. They bind to WNT response elements (WREs) in the genomic region of target genes involved in cell proliferation, survival, and migration [7], [19]. In the context of the intestinal epithelium, the β-catenin/Tcf4 complex regulates the expression of genes involved in the development and proliferation of normal and malignant epithelia [20], [21]. β-catenin, however, forms complexes with other transcription factors, including nuclear hormone receptors [22], [23]. This interaction modulates the transcriptional activity of the partners, depending on the specific tissue or nuclear receptor [24]–[28]. Our previous studies on the relationship between WNT and TRα1, combined with these observations, compelled us to investigate the physical interaction between TRα1 and β-catenin, the eventual involvement of Tcf4 in the complex, and its physiopathological relevance.

We established that the increased levels of the β-catenin/Tcf4 complex affects the transcriptional activity of TRα1 *in vivo*. We show that TRα1 interacts with the β-catenin/Tcf4 complex in the nuclei of Caco2 cells and that this interaction strongly reduces TRα1 functionality, but has a positive effect on the WNT downstream response *in vitro*. Finally, we observed the recruitment of TRα1 on the WRE regions in pre-cancerous and cancerous intestinal lesions.

## Results

### The expression of TRα1 direct target genes is impaired in *vil*-TRα1/Apc mice

We analyzed the expression profile of TRα1 target genes in normal mucosae or tumors from mice of different genotypes to gain additional insights on the cross-regulation between TRα1 and WNT pathways in gut tumorigenesis. Six-month-old *vil*-TRα1 [9], Apc^+/1638N^ [29] and double-mutant *vil*-TRα1/Apc [9] mice were analyzed. The *vil*-TRα1 mice are characterized by hyperproliferation in the intestinal crypts and a low rate of adenoma development in the small intestine and colon [9]. The Apc^+/1638N^ develop a small number of adenocarcinomas, starting at approximately six months of age; these tumors occur primarily in the small intestine [29], [30]#. The *vil*-TRα1/Apc mice develop adenocarcinomas in the small intestine and colon at a higher frequency than do the Apc mutants. Moreover, the tumor appearance and progression to invasiveness are also accelerated in these mice. Finally, WNT activity in the tumors of these animals is increased compared with Apc mutants [9].

We compared the expression profiles of *Ctnnb*1 and *Sfrp2*, TRα1-direct target genes [15], [16], and of *Ccnb1 and Cdc2a*, TRα1-indirect target genes [16]. For *Ctnnb1* and *Sfrp2*, we observed an increased mRNA levels in the *vil*-TRα1 mice compared with the WT mice, while in the normal mucosa or tumors of the Apc mice, the mRNA levels slightly decreased (*Ctnnb1*, Figure 1A) or did not change (*Sfrp2*, Figure 1B). However, in the *vil*-TRα1/Apc mice, the up-regulation of both genes was blunted, and the mRNA level unchanged (*Ctnnb1*, Figure 1A) or decreased (*Sfrp2,* Figure 1B) in the tumors. When we examined the TRα1-indirect target genes *Ccnb1* and *Cdc2a*, we observed that TRα1 overexpression stimulated the mRNA levels of these genes independently of the Apc mutation (Figure 1C, D). We also analyzed the *Ctnnb1* and *Sfrp2* mRNA expression in one-month-old animals. In fact, the tumorigenic program triggered by the loss of Apc heterozygosis [30] at that age is not yet accomplished, and the *vil*-TRα1/Apc mice do not yet show any signs of mucosal alteration. Interestingly, the mRNA expression level of TRα1-direct target genes in these animals was comparable with that of the *vil-*TRα1 mice, and in both cases, significantly higher than in the WT intestine (Figure S1A, B). We excluded the fact that the TRα1-reduced transcriptional activity is due to a lower availability of hormones, as the circulating TH level is not altered in the animals of different genotypes [9]. However, the intracellular concentration of TH may depend on T3 and T4 metabolism, which is locally regulated by the iodothyronine deiodinase selenoenzymes (Dio1, Dio2 and Dio3) [31], [32]. Next, we considered the possibility that the transcriptional activity of TRα1 was reduced by local hypothyroidism within the tumors and checked the levels of the three enzymes. However, when we analyzed the expression of the Dio mRNAs, we observed that only Dio1 was expressed, and its levels did not change in the intestine of different genotypes or in the tumors (Figure S1C), confirming that the cellular context was not hypothyroid. It is worth noting that in another context, Dio1 has been shown to be TH-responsive [31]; however, this difference may be due to the well-described tissue-specific regulation of TH target genes [10].

**Figure 1:** Analysis of TRα1 target genes in mice of different genotypes. RT-qPCR experiments were performed in the intestine of 6-month-old mice of the indicated genotype to analyze the mRNA levels of *Ctnnb1* (A), *Sfrp2* (B), *Ccnb1* (C) and *Cdc2a* (D). Values represent fold change ± sd after normalization to the wild-type [WT] animals. *: P<0.05, **: P<0.001, compared with the WT; #: P<0.05, ##: P<0.01 compared with the *vil*-TRα1 animals, by two-tailed Student's t-test (n = 4). N, normal mucosa; T, tumor.

### The Wnt3a ligand is not sufficient to affect TRα1 transcriptional activity in an ex vivo assay

We used intestinal epithelial primary culture to evaluate whether activation of the WNT pathway by an agonist could impair TRα1 transcriptional activity. To selectively modulate TRα1 and WNT, we treated the cells with T3 and the canonical Wnt3a ligand [33] alone or in combination. We observed that T3 and/or Wnt3a increased the number of proliferating cells (Figure 2A) and expressing nuclear β-catenin [Figure 2B]. The increase of both activated β-catenin protein level (Figure 2C) and *Ccnd1* mRNA expression (Figure 2D), indicated that the cells were responding to the simple treatments as previously shown [15], [34]. When we investigated the expression of *Ctnnb1* and *Sfrp2*, TRα1 direct target genes, both mRNA levels increased upon T3 treatment, as expected. Wnt3a had no effect on *Ctnnb1* mRNA (Figure 2E) but stimulated *Sfpr2* mRNA (Figure 2F). Finally, when the cells were treated with Wnt3a and T3, the TRα1 targets behaved as they did when treated only with T3, because they were not affected by the co-treatment with Wnt3a (Figures 2E, F). The expression of TRα1 or Tcf4 was not altered by T3 alone or in combination with Wnt3a (not shown).

**Figure 2:** The Wnt3a ligand is not sufficient to impair TRα1 transcriptional activity ex vivo. The primary cultures of intestinal epithelial cells were treated with 10 ng/ml of Wnt3a and/or 10^−7^ M of T3 for 24 hours. (A) The number of proliferating cells in the different experimental conditions was analyzed by Ki67 immunolabeling; all of the nuclei were labeled by Hoechst. The percentage of Ki67-positive nuclei was determined by counting under a fluorescence microscope (Zeiss Axioplan). The histograms represent the summary (mean ± sd) of the scoring of specific immunolabeling in two independent experiments each conducted in triplicate (n = 50). (B, C) Analysis of β-catenin in intestinal epithelial primary cultures by immunolabelling (B) and WB (C). Cells were in control, T3, Wnt3a and T3+Wnt3a conditions as indicated. Pictures in B show the fluorescent staining of the nuclei (blue), β-catenin (red) and the merging of each simple labeling. Bar: 15 µm. For the WB (C), we used a specific antibody allowing the detection of activated non-phosphorylated β-catenin [54], [55]. Actin was used as loading control. The image is representative of two independent experiments. Each lane represents whole protein extracts (50 µg/lane). (D–F) RT-qPCR analysis to evaluate mRNA levels of *Ccnd1*, *Ctnnb1* and *Sfrp2*. Results are from three independent experiments, each conducted in duplicate. Values represent fold change ± sd after normalization to the control condition (Ctrl). *: P<0.05, **: P<0.01, ***: P<0.001 by two-tailed Student's t-test (n = 6).

### *Tcf7l2* (Tcf4) is overexpressed in *vil-*TRα1/Apc mice

The data obtained using the *in vitro* and *in vivo* approaches strongly suggested that β-catenin stabilization induced by Wnt3a is not sufficient to impair TRα1 transcriptional activity. Thus, the hypothesis that an increased level of both β-catenin and Tcf4 could affect TRα1 functionality was tested. We examined the mRNA expression of Tcf4 in the normal intestine and tumors from animals of different genotypes. The Tcf4 mRNA expression in *vil*-TRα1 or the normal mucosa of Apc mice was similar to that of WT animals (Figure 3A). However, the mRNA level significantly increased in the normal mucosa of the *vil*-TRα1/Apc mice and was even further upregulated in the tumors. We also observed an increased level of Tcf4 mRNA in the lesions from Apc mice compared with the healthy mucosa (Figure 3A). This trend was different from that observed for *Lef1* mRNA, another transcriptional partner of β-catenin in the intestine [35], [36]. In fact, *Lef1* mRNA level was significantly increased only in the lesions independently of the animals' genotype (Figure 3B).

**Figure 3:** Analysis of *Tcf7l2* (Tcf4) and Wnt target genes in mice of different genotypes. RT-qPCR experiments were performed in the intestine of 6-month-old mice of the indicated genotype. (A) Tcf4, (B) *Lef1*, (C) *c-Myc* and (D) *Ccnd1* mRNA levels were analyzed. Values represent fold change ± sd after normalization to wild-type (WT) animals. *: P<0.05, **: P<0.01 compared with the WT; $: P<0.05, $$: P<0.01 compared with the healthy mucosa of the same genotype; @: P<0.05, @@: P<0.01 compared with *vil*-TRα1/Apc N and T; #: P<0.05 compared with *vil*-TRα1, by two-tailed Student's t-test (n = 4). N, normal mucosa; T, tumor.

Finally, we analyzed the expression of *Ccnd1* and *c-Myc*, the WNT target genes, and we observed their significant upregulation in the *vil-*TRα1 and in the normal mucosa of *vil-*TRα1/Apc mice compared with that of the WT or the normal mucosa of Apc mice [Figure 3C, D], in accordance with our previous results [9]. The expression level of these WNT target genes significantly increased in the tumors of both genotypes compared with the respective normal mucosae (Figure 3C, D).

### The β-catenin/Tcf4 complex interferes with TRα1 functionality in vitro

The data described above strongly suggested that a negative feedback loop could occur between TRα1 and the β-catenin/Tcf4 complex. To test this hypothesis, we used a luciferase reporter system containing a synthetic tandem of TR-binding sites organized as DR4 (DR4-luc) [15] and monitored its response upon β-catenin and/or Tcf4 transfection. These experiments were performed in Caco2 cells maintained in T3-depleted serum with and without the addition of a supra-physiological concentration of T3 (Figure 4A). In the control condition, we observed a strong and significant increase in luciferase activity upon T3 treatment due to the presence of endogenous TRα1. It is worth noting that we observed a response to T3 addition in all conditions analyzed (Figure 4A). The transfection of β-catenin alone did not affect the DR4-luc response to the endogenous TRα1 stimulated by T3, while Tcf4 alone slightly reduced the reporter activity. Interestingly, Tcf4 in combination with β-catenin significantly reduced the T3 response of the endogenous TRα1 compared with the control (Figure 4A). As expected, the TRα1 transfection in the cells treated with T3 significantly enhanced the luciferase activity in comparison with the control (Figure 4A). This T3-mediated response in TRα1-transfected cells was slightly reduced in the presence of β-catenin, significantly decreased in the presence of Tcf4 and a stronger negative effect was observed by combining Tcf4 and β-catenin co-transfection.

**Figure 4:** β-catenin/Tcf4 complex interferes with TRα1 functionality in luciferase assay in vitro. (A) The DR4-luc luciferase reporter was transfected into Caco2 cells maintained in T3-depleted serum with or without supplementation with T3 as indicated, together with TRα1, Tcf4 or β-catenin expression vectors in different combinations. (B, C) The DR4-luc luciferase reporter (B) or TopFlash luciferase reporter (C) was transfected into Caco2 cells maintained in culture medium containing physiological concentrations of T3, together with the β-catenin/Tcf4 complex in the presence or absence of the TRα1 expression vector. Histograms represent mean ± sd from three independent experiments, each conducted in triplicate (n = 9). *: P<0.05, **: P<0.01 compared with the control condition (Ctrl); #: P<0.05, ##: P<0.01, compared with the TRα1 condition; $: P<0.05 compared with the TRα1+β-catenin condition; ££: P<0.01 compared with the β-catenin or β-catenin+Tcf4 condition, by two-tailed Student's t-test.

We also measured the DR4-luc activity in cells maintained in culture medium containing physiological concentrations of T3 [37] (Figure 4B). As expected, TRα1 transfection significantly induced the luciferase activity compared with the control. Moreover, this response was impaired by co-transfection of TRα1 with the β-catenin and Tcf4 vectors. The luciferase activity induced by TRα1 overexpression was not affected by β-catenin alone but was slightly reduced by Tcf4 (Figure 4B). We decided to verify if these combinatory transfections could also affect the activity of the WNT-reporter system TopFlash, which responds to the β-catenin/Tcf complex [38]. We observed a significant increase of TopFlash activity when TRα1 was transfected together with β-catenin or Tcf4 compared with the simple β-catenin or Tcf4 conditions (Figure 4C). We observed a slight up-regulation of the TopFlash activity, marginally significant, when TRα1 was transfected together with β-catenin/Tcf4. We verified the specificity of these responses by using mutated DR4-luc or FopFlash reporters (data not shown).

### TRα1 binding on chromatin changes during gut tumorigenesis

Our findings strongly indicated that the increased level of the β-catenin/Tcf4 complex significantly reduced the TRα1 transcriptional activity both in cell lines and *in vivo*. To define the mechanism involved, we evaluated whether TRα1 could physically interact with β-catenin and/or Tcf4, as has been shown for other nuclear receptors [22], [23]. For this purpose, a co-immunoprecipitation (Co-IP) approach was employed to selectively target the endogenous proteins in the nuclei of Caco2 cells. After validating that TRα1 and β-catenin interact specifically in cell nuclei (Figure S2), we also analyzed the involvement of Tcf4. Interestingly, we observed that in the nuclei of the Caco2 cells the endogenous TRα1 is associated with β-catenin (Figure 5, upper and middle panels) as well as with Tcf4 (Figure 5, upper and lower panels). Moreover, all these interactions do not depend on T3 levels.

**Figure 5:** Physical interaction between TRα1 and the β-catenin/Tcf4 complex. Nuclear extracts from Caco2 cells, maintained in T3-depleted (−) or T3-supplemented (+) serum, were immunoprecipitated with antibodies directed against endogenous Tcf4, β-catenin or TRα1 and analyzed by WB by using the antibodies as indicated. Rabbit IgG was used as negative control. Ponceau red was used as whole-protein (50 µg/lane) loading control. Histone H1 was used to check the enrichment and was the loading control for the nuclear proteins in the inputs. The pictures are representative of at least three independent experiments.

We then investigated the presence of the three proteins on the chromatin, by using an *in vivo* chromatin immunoprecipitation (ChIP) approach to analyze the TREs and WREs of the specific target genes of TRα1 and WNT, respectively. The ChIP assay was performed on WT intestine and the normal mucosa or tumors from *vil*-TRα1/Apc mice using anti-TRα1, anti-Tcf4, anti-β-catenin antibodies or rabbit IgG (as negative control). As shown in Figures 6A and S3A, in the WT intestine, TRα1 binds to the promoter region of the *Sfrp2* gene, which contains the TRE [16]; however, there was no recruitment of the β-catenin/Tcf4 complex independently of the genotype or the pathological condition (Figures 6A and S3A). This result was similar to that obtained by an *in vitro* EMS assay in which TRα1 binds to a DR4 element without forming a complex with β-catenin and/or Tcf4 (Figure S4). As the *Sfrp2* expression profile suggested, the TRα1 chromatin occupancy changed between the WT and mutant intestine. In fact, in *vil-*TRα1/Apc mice, the TRα1-specific-DNA binding on the promoter was lost compared with the WT animals (Figures 6A and S3A). We confirmed this same profile of TRα1 chromatin occupancy on the *Ctnnb1* TRE [15] (Figures 6B and S3B).

**Figure 6:** Chromatin occupancy of TRα1, β-catenin and Tcf4 on genomic regions of target genes. ChIP analysis was performed with chromatin isolated from the intestine of WT or *vil*-TRα1/Apc mice (healthy mucosa and tumor) and immunoprecipitated with anti-TRα1, anti-β-catenin, anti-Tcf4 antibodies or rabbit IgG (negative control). qPCR was performed using specific primers covering the TRE of *Sfrp2* (A) and *Ctnnb1* (B), the WRE of *Axin2* (C) and c-*Myc* (D) or the promoters of *Villin* (E) and *36B4* (F); the *Ppia* gene was used as internal control. Data are representative of one of two experiments. Histograms represent the specific-DNA enrichment in each sample immunoprecipitated with the indicated antibody. The black bar in A–D delineates the threshold of binding specificity determined by the IgG non-specific binding. N, normal mucosa; T, tumor.

Next, we analyzed the specific DNA binding of Tcf4 and β-catenin on their target genes and the eventual presence of TRα1 in the same regions. A WRE has been described within the *Axin2* promoter [39]. We observed that the Tcf4 occupancy on this promoter was similar in the different experimental conditions (Figures 6C and S3C) and that the presence of β-catenin on the WRE increased during tumorigenesis. More interestingly, TRα1 was not present on the *Axin2* WRE region in the WT intestine but was clearly enriched on it, both in normal mucosae and the tumors of *vil*-TRα1/Apc mice (Figures 6C and S3C). We confirmed a similar trend of TRα1 binding on the WRE region of *c-Myc*, another classical direct WNT target [40] (Figures 6D and S3D), while no specific binding was detected on the *Villin* or *36B4* gene promoters (Figures 6E,F and S3E,F). Given the intriguing result of TRα1 binding to WRE regions, we used the software NUBISCAN (http://www.nubiscan.unibas.ch) to search for the presence of putative nuclear receptor binding sites *in silico*. No TREs were found within the *Axin2* or *c-Myc* genomic regions containing the WREs analyzed (data not shown).

## Discussion

The process of intestinal maturation and its homeostatic control by TH-TRα1 in mice results from a complex modulation of genes and signaling pathways, including the WNT, Notch and BMP [16]. The WNT pathway is considered a major signaling modulator of the physiological and pathological cell proliferation in the intestinal epithelium [41]#. Moreover, due to its direct action on epithelial stem cells, this pathway is also a main regulator of epithelial homeostasis [41]. Interestingly, the superfamily of the Nuclear Hormone Receptors (NHR), to which TRα1 belongs, displays several levels of functional and physical interactions with the WNT pathway [22], [23]. Although this interaction is relatively conserved among NHRs, there are however several differences. Some NHRs, such as VDR, PPARγ, and AR, are found in a complex with both β-catenin and Tcf/Lef, while others, such as ER and AR, can be found in a complex with Tcf/Lef in the absence of β-catenin [42]–[46]. The functional outcomes of these protein-protein interactions can also differ depending on the NHR. Generally speaking, β-catenin synergistically activates NHR activity, and NHR reciprocally deactivates or even represses β-catenin activity [22], [23]. This effect can be attributed to a large number of mechanisms involving E-cadherin expression, the competition between Tcf/Lef and NHRs for binding to β-catenin and/or p300 or the recruitment of co-repressors such as TLE, NCoR, and SMRT [22], [23]. However, these interactions are highly dependent on the cellular context and can create divergent effects. For example, PPARγ, whose expression and activity is negatively regulated by WNT in mesenchymal stem cells, undergoes positive regulation of the WNT signal in colon cancer cells [45]. A similar phenomenon is reported for VDR, which super-activates β-catenin activity in keratinocytes [42]#, but attenuates it in colorectal cancer [25], [28], [47]. In this context, the physical interaction between TRα1 and the transcriptional effectors of WNT was an attractive field of investigation. In fact, it had been previously shown that TRβ1 and β-catenin can interact directly to form a complex in thyrocytes [24]. This study, however, did not define the involvement of Tcf4 or the effect on TRβ1 activity. In this study, we have provided the first evidence that TRα1 interacts with β-catenin. Moreover, this interaction also involves Tcf4. There are two major differences between the interaction of TRα1/β-catenin/Tcf4 in the intestinal epithelium and that of TRβ1/β-catenin in thyrocytes. The first is the destabilization of the TRβ1/β-catenin complex by the hormone T3 [24], while we found no evidence for any T3-mediated effect on TRα1/β-catenin/Tcf4. The second is the action of the complex on the WNT pathway. In fact, TRβ1 induces the degradation of β-catenin [24], but TRα1 stabilizes it and activates WNT [9], [15]. It is worth noting that TRα1 and TRβ1 often play opposite roles [5], [48], and differences in the cell context may also explain these divergences.

Previously, we described several levels of complex relationships between WNT and the TRα1 pathways [10]#. First, we showed that TRα1 induces WNT activation and enhances cell proliferation [15], [16]. Second, we demonstrated a synergy between these two pathways during the process of intestinal tumorigenesis [9]. Finally, the third level of regulation outlined herein validates the positive action of TRα1 on WNT through a protein-protein interaction. In light of these new results, we propose that an intriguing feedback loop can also occur and that WNT over-activation likely decreases TRα1 transcriptional activity (proposed model of action in Figure 7). However, from our results, we cannot definitively conclude that this protein-protein interaction involves only the three partners we analyzed, as other factors that have not yet been identified may also participate in the complex.

**Figure 7:** Proposed molecular model for the action of TRα1 in controlling the WNT signaling pathway in the intestine. In physiological conditions (WT), TRα1 binding on TREs positively regulates the expression and stabilization of β-catenin, and then contributes to maintaining tissue homeostasis. In *vil*-TRα1 mice, there is an increased level of β-catenin expression and stabilization that leads to WNT activation and hyper-proliferation. In *vil-*TRα1/Apc mice, the stronger β-catenin stabilization and Tcf4 overexpression might be responsible of the shift in TRα1 binding from TREs to WREs. The physical interaction between TRα1 and β-catenin/Tcf4 we showed can explain its presence on the WREs. We speculate that this is a novel mechanism of WNT induction promoting the activation and/or the acceleration of the tumorigenic process. TREs, Thyroid hormone response elements; WREs, WNT response elements. Solid lines indicate genomic actions; dotted lines represent the speculative model of a negative regulatory loop involving non-genomic actions and eventually other(s) factor(s). Double black arrows indicate crypt width in WT and *vil*-TRα1 intestinal sections.

It has been shown that the functional interactions between signaling pathways involved in gut homeostasis can have a primary importance in the process of cell transformation. This is the case, for instance, of the synergy between WNT and Notch [49] or WNT and TRα1 [9]. In both examples, Notch and TRα1 induce increased cell proliferation, which is likely to determine an early mutagenic event in the Apc gene, and finally an acceleration of the tumorigenic process. We have shown that TRα1 interacts with the β-catenin/Tcf4 complex and speculate that this interaction might play a key role during the process of intestinal tumorigenesis by stabilizing the WNT effectors on their target genes. We could not observe, however, a clear-cut difference in the expression level of the WNT targets in the adenocarcinoma of different genotypes. One possibility is that once the tumoral program is completed, the molecular differences may be less apparent at the mRNA level. In addition, colon cancer is genetically heterogeneous and is composed of distinct subpopulations [50], [51]. Hence, interpretation of results from a comparative gene expression analysis in whole tumors can be hampered by such heterogeneity. In support of both assumptions, an upregulation of the WNT targets in the normal mucosa of the *vil-*TRα1/Apc mice is evident and might play a critical role during the early steps of gut tumorigenesis. With regard to the direct targets of TRα1, the overexpression of β-catenin/Tcf4 clearly inhibits their TRα1-dependent upregulation, but it does not affect the expression of the TRα1 indirect targets *Ccnb1* and *Cdc2a*. It is probable that other transcription factors and compensatory mechanism(s) occurring *in vivo* may also be responsible for their expression levels.

Our results suggest that the binding of TRα1 to its DNA targets is shifted to the WNT targets when the β-catenin/Tcf4 protein levels increase (Figure 7). This condition is typical of intestinal cancers characterized by mutations in components of the WNT pathway (including *Apc*, *Ctnnb1* and *Axin2*) 50,52 that allow for β-catenin increase and stabilization. With regard to Tcf4 expression, we observed its upregulation in the tumors of both Apc and *vil*-TRα1/Apc mice. Interestingly, we also observed an increased expression of Tcf4 in the normal mucosa of the *vil*-TRα1/Apc mice but not in the normal mucosa of the Apc animals. Taken together, our previous and present data strongly suggest that even if we refer to “*vil*-TRα1/Apc mice normal mucosa”, this may only be indicative of the morphological appearance. Indeed, from a molecular standpoint, it differs in several ways from the WT mucosa [9] (this paper) and clearly indicates an altered pre-cancerous status.

In conclusion, we have shown that in the context of intestinal lesions, TRα1 reshapes its function and induces specific genomic and non-genomic events. TRα1 transcriptional activity was negatively modulated by increased levels of β-catenin/Tcf4 and the binding to its target genes was also impaired. Interestingly, TRα1 was recruited to WNT target genes specifically within the lesions. This dual mechanism can have important repercussions and opens a new perspective in studying the sequential events of tumor development. An obvious speculation is that β-catenin/Tcf4 activity on their target genes could be reduced in the absence of TRα1. Our preliminary results from TRα^0/0^/Apc mice sustain this assumption (our unpublished observations); however, it is necessary to further confirm this result to account for the delay in or absence of tumor formation in these animals. A future challenge will be to define how complex cross-regulation and integrated networks, such as those involving the NHR and WNT pathways, can affect the cellular phenotype when signals are altered. These data will surely be of importance for translational research and could help explain the contradictory results concerning NHRs and carcinogenesis.

## Materials and Methods

### Animals and sample collection

We used *vil*-TRα1, *vil*-TRα1/Apc, Apc^+/1638N^ and wild-type animals [9]. Mice were housed and maintained with approval from the animal experimental committee of the Ecole Normale Supérieure de Lyon (Lyon, France) and in accordance with European legislation on animal care and experimentation. Lyon University's “Comité d'Evaluation Commun au Centre Léon Bérard, à l'Animalerie de transit de l'ENS, au PBES et au laboratoire P4” (CECCAPP) and the “the Comité Régional d'Ethique pour l'Expérimentation Animale» (CREEA) approved all animal studies (agreement no. 0230). Animals were sacrificed, and the intestine (normal mucosae and tumors) was quickly removed. We recovered tumors and normal portions of the mucosa under a binocular microscope (Olympus) and froze them in liquid nitrogen for RNA extraction or the ChIP assay.

### Intestinal epithelium primary cultures, immunolabelling and western blot

Intestinal epithelial primary cultures were derived from 4–6 day old neonatal mice according to Evans and colleagues [53]. Briefly, after sacrifice, the entire small intestine was removed. The epithelium was isolated as intact organoids by enzymatic dissociation using collagenase type XI (Sigma) and dispase (Boehringer Mannheim), followed by physical disaggregation and filtration on gauze. Organoids were plated in Dulbecco's modified Eagle medium (DMEM, Invitrogen) supplemented with 2.5% heat-inactivated fetal calf serum (Gibco), 20 ng/ml epidermal growth factor (Sigma), and insulin-transferrin-selenium diluted 1/100 (Sigma). Culture surfaces were coated with Matrigel™ Basement Membrane Matrix (BD Biosciences). For immunolabeling experiments, cover-slips were inserted in the wells before coating. For proliferation studies, 10 µM BrdU was added to the culture medium for an overnight incubation. The purity of the epithelial colonies was analyzed by immunolabeling for specific markers: epithelial cells: anti-cytokeratins (ICN); fibroblasts: anti-vimentin (Sigma); smooth muscle cells: anti-smooth muscle actin (Sigma). For treatment experiments, after 2 days of culture, the vehicle alone or 10^−7^ M T3 and/or 10 ng/µl of recombinant Wnt3a (R&D system) was added to the culture medium for 24 hours.

Immunolabeling was performed on 2% paraformaldehyde-fixed cultures, as previously described by Rezza and colleagues [32]. We used anti-Ki67 (Labvision MBL) and anti-β-catenin (Santa Cruz) primary antibodies.

Western blot (WB) was performed on whole-protein extracts obtained by homogenizing the samples in RIPA buffer, as described in [32]. Whole protein extracts (50 µg/lane) from cells maintained in the different experimental conditions were analyzed. We used anti-activated β-catenin (Upstate) and anti-actin (Sigma).

### Cell lines and transfection experiments

This study was performed on the human Caco2 colorectal cancer cell line (from the American Type Culture Collection). Caco2 cells (50,000 cells/well in 24 multiwell plates) were cultured in DMEM supplemented with 10% heat- inactivated fetal calf serum. We used the following vectors: pGl2-DR4-Luc and pGl2-mutDR4-Luc (200 ng/well) and pGS5-TRα1 [15] (100 ng/well); TopFlash and FopFlash (Upstate; 200 ng/well); pCIneo-b-cateninXL (100 ng/well), Evr2-Tcf4E (100 ng/well; kind gift of Professor Waterman, UC Irvine, USA); pRL-CMV (1 ng/well; Promega). The vectors were transfected using the Exgen transfection reagent (Euromedex). For the T3 treatments, the cells were maintained in thyroid hormone-depleted serum [35]. T3 (10^−6^ M) or vehicle alone was added to the culture medium 24 hours before the end of the culture. Luciferase activity was measured 48 hours after transfection using the luciferase dual system (Promega).

### Coimmunoprecipitation assay and western blot analysis

Coimmunoprecipitation (CoIP) studies were conducted on Caco2 cells using a slightly modified procedure described by Guigon and colleagues [24]. Nuclear and cytoplasmic extracts were pre-cleared with Protein A magnetic beads (Invitrogen) for 4 hours at 4°C. Immunoprecipitations of endogenous complexes were conducted overnight at 4°C with anti-Tcf4 (Santa Cruz), anti-β-catenin (Santa Cruz), anti-TRα1 [15] antibodies. As negative controls, the extracts were incubated with rabbit IgG (Promega). The complexes were washed and then recovered with Protein A magnetic beads. Immunoprecipitated proteins were subjected to SDS-PAGE and western blot analysis by using the different antibodies mentioned above. Whole proteins (50 µg/lane) on the blots were stained with Ponceau red. The nuclear extracts and loading in inputs were examined by using an anti-Histone H1 antibody (Santa Cruz).

### RNA extraction and RTqPCR analysis

RNA was extracted from tissue samples using the Qiagen RNeasy Kit (Qiagen). To avoid the presence of contaminating DNA, DNase digestion was performed on all preparations. Reverse transcription was performed using MuMLV reverse transcriptase (Promega) on 1 µg of total RNA using random hexanucleotide priming (Promega) according to the manufacturer's instructions. For the primary cultures, RNA was extracted using the Absolutely RNA Nanoprep Kit (Stratagene). Reverse transcription was performed using the SuperScript III First-Strand Synthesis SuperMix for qRT-PCR (Invitrogen) on 300 ng of total RNA. All of the cDNA samples were purified using the Qiagen PCR Purification Kit (Qiagen) before use for the qPCR experiments. The qPCR was performed with SYBR green PCR master mix (Qiagen) in an MxP3000 apparatus (Stratagene). The data from the qPCR were normalized to 36B4 levels for each sample. The primers are listed in Table S1A.

### Electrophoretic mobility shift assay (EMSA)

Tcf4, β-catenin, TRα1 and RXRα full-length cDNAs were transcribed/translated in vitro using the quick TNT kit (Promega) according to the manufacturer's protocol. We performed the EMSA assay on the DR4-radiolabeled probe, as previously described [18], in a buffer similar to that of the CoIP: 3% glycerol, 20 mM HEPES, 3 mM DDT, 0.3% NP40, 100 mM KCl, protease inhibitor cocktail (Roche), 4 mM spermidine, and poly-dI-dC (1.5 µg). Where indicated, anti-TRα1 [15] and anti-Tcf4 (Santa Cruz) antibodies were included in the reaction mix.

### Chromatin immunoprecipitation (ChIP)

The ChIP study was performed on 10 mg of samples collected from the intestine of *vil*-TRα1/Apc (healthy mucosa and tumors) and WT mice. The samples were minced with a razor blade and crosslinked with 1% formaldehyde at room temperature for 15 minutes. The crosslinking reaction was stopped by the addition of glycine to a final concentration of 0.125 M, and the samples were incubated at room temperature for 5 minutes. The samples were then centrifuged at 200 g to pellet the pieces. The fragments were washed once in cold PBS containing protease inhibitor cocktail (Roche) and then disaggregated by 10 strokes in a Dounce homogenizer. The resulting homogenate was centrifuged at 2000 g, the pellet recovered was then incubated in SDS buffer (1% SDS, 50 mM TRIS pH 8.1, 10 mM EDTA) on ice for 10 minutes. After 15 minutes of sonication (30 sec on/30 sec off cycles, Biodisruptor), the samples were centrifuged at maximum speed at 4°C, and the supernatant was recovered and quantified by Nanodrop (ND-1000 UV-Vis Spectrophotometer, NanoDrop Technologies). The same amount of each sample was diluted 1∶10 in dilution buffer (0.01% SDS, 1.1% Triton X-100, 1.2 mM EDTA, 16.7 mM Tris-HCl, pH 8.1, 167 mM NaCl). After pre-clearing with Protein A magnetic beads (Invitrogen), each sample was divided into four samples, and the precipitation was performed using 9 µg of each antibody (anti-Tcf4, Santa Cruz; anti β-catenin, Santa Cruz; anti-TRα1 [15] or rabbit IgG). At the end of the reaction and washing steps, the complexes were recovered using protein A magnetic beads. The DNA was extracted after Proteinase K (Fermentas) and phenol-chloroform treatments. Specific DNA fragments were analyzed by qPCR using a SYBR green PCR master mix (Qiagen) in an MxP3000 apparatus (Stratagene). The primers designed to amplify the genomic regions containing: 1) TREs we previously described [15], [16]; 2) WREs described in literature [39], [40]; and 3) the *villin* and *Rplp0* (*36B4*) promoters, as negative controls [15]. Primer sequences are listed in Table S1B; the *Ppia* gene was used in all reactions as internal control.

## Supporting Information

Figure S1 **RT-qPCR analysis in mice.** (A, B) Analysis of TRα1-direct target genes in 1 month-old WT, *vil*-TRα1 and *vil*-TRα1/Apc mice. RT-qPCR analysis was performed to evaluate the mRNA levels of Ctnnb1 and Sfrp2. Values represent fold change ± sd after normalization to the wild-type (WT) animals. *: P<0.05, **: P<0.01 compared with the WT by two-tailed Student's t-test (n = 4). (C) Analysis of iodothyronine deiodinase selenoenzyme type 1 (Dio1) mRNA expression in WT, *vil*-TRα1, Apc and *vil*-TRα1/Apc mice. RT-qPCR experiments were performed in the intestine of 6-month-old mice. Values represent specific mRNA expression ± sd after normalization to 36B4 (n = 4). N, normal mucosa; T, tumor.
(PDF)

Figure S2 **Physical interaction between TRα1 and the β-catenin in nuclei.** Cellular lysates from Caco2 cells, maintained in T3-depleted (−) or T3-supplemented (+) serum, were fractionated into nuclear (N) and cytoplasmic (C) extracts. Lysates were immunoprecipitated with antibodies directed against endogenous β-catenin (upper panel) or TRα1 (lower panel), and the WB analysis of the indicated proteins was performed. Rabbit IgG was used as negative control. Ponceau red was used as whole-protein (50 µg/lane) loading control. Histone H1 was used to check the enrichment and was the loading control for the nuclear proteins in the inputs. The pictures are representative of at least three independent experiments.
(PDF)

Figure S3 **Chromatin occupancy of TRα1, β-catenin and Tcf4 on genomic regions of target genes.** ChIP analysis was performed with chromatin isolated from the intestine of WT or *vil*-TRα1/Apc mice (healthy mucosa and tumor) and immunoprecipitated with anti-TRα1, anti-β-catenin, anti-Tcf4 antibodies or rabbit IgG (negative control). qPCR was performed using specific primers covering the TRE of Sfrp2 (A) and Ctnnb1 (B), the WRE of Axin2 (C) and c-Myc (D) or the promoters of Villin (E) and 36B4 (F); the Ppia gene was used as internal control. Histograms represent the specific-DNA enrichment in each sample immunoprecipitated with the indicated antibody. The black bar in A–D delineates the threshold of binding specificity determined by the IgG non-specific binding. N, normal mucosa; T, tumor.
(PDF)

Figure S4 **Electromobility Shift Assay on DR4 response element.** (A) EMSA analysis was performed to examine the TRα1/β-catenin/Tcf4 complex formation on a DR4-radiolabeled probe. In vitrotranscribed/translated proteins were added to the mixture as indicated, and the DNA-protein complexes were separated by native gel electrophoresis. Specific antibodies were added to assess the protein[s] involved in the complex. In all of the conditions, only TRα1 alone binds to the labeled probe. (B) EMSA performed in the presence of the TRα1 transcriptional partner RXRα. It is worth noting that even in the presence of RXRα, there is no β-catenin/Tcf4 binding to TRα1 on a TRE.
(PDF)

Table S1 (A) Oligonucleotides used for the RT-qPCR study. (B) Oligonucleotides used for qPCR study after ChIP assay.
(PDF)
